# The Experimental Exploration of TCM Theory “Treating the Same Disease with Different Approaches” on an Ulcerative Colitis Model

**DOI:** 10.1155/2022/4916540

**Published:** 2022-06-30

**Authors:** Lulu Ni, Lingzhong Kong, Yajun Tang, Yangfan Nie, Xinyue Wang, Xue Yang, Li Zhu, Shan Jing

**Affiliations:** ^1^Department of Basic Medicine, Jiangnan University, Wuxi, Jiangsu 214122, China; ^2^Department of Rehabilitation Acupuncture Medicine, Bozhou People's Hospital, Bozhou, Anhui 236800, China; ^3^Department of Gastroenterology, Ningbo Municipal Hospital of Traditional Chinese Medicine, Ningbo, Zhejiang 315016, China; ^4^Department of Internal Medicine of TCM, Dong-Zhimen Hospital, Beijing University of Chinese Medicine, Beijing 100700, China; ^5^Department of Internal Medicine of TCM, Hennan University of Traditional Chinese Medicine, Zhengzhou, Henan 450003, China; ^6^Department of Internal Medicine of TCM, Nantong Hospital of Traditional Chinese Medicine, Nanjing University of Chinese Medicine, Nantong, Jiangsu 226000, China

## Abstract

There is a relationship between lung injury and ulcerative colitis. Currently, traditional Chinese medicine (Huangqi Jiegeng (HQJGD) and Huangqi Huanglian decoctions (HQHLD)) is commonly used for UC-related lung injury; however, the mechanisms of these drugs remain unclear. In this study, UC models were established with the mucous membrane of colon allergize combined with TNBS-alcohol enteroclysis for 4 weeks. The pathological changes in the lung, intestine, liver, and kidney were observed; cytokines, chemokines, and adhesion molecules in lung tissue were detected in order to explore the immunological mechanism of UC-related lung injury and the intervention mechanism of traditional Chinese medicine in treating the lung and intestine in the immune-TNBS-ethanol rat model. Histology examinations demonstrated evident pathological changes in the lungs and intestines of the model groups. Furthermore, all groups treated with TCMs demonstrated reduced expressions of toll-like receptor 4, nuclear factor kappa-B, and macrophage migration inhibitory factor. Additionally, radioimmunoassay and immunohistochemistry showed tumor necrosis factor-*α*, interleukin-6, and 8 expression downregulation. The results showed that HQJGD and HQHLD could alleviate pulmonary inflammation in UC-related lung injury by obviously improving the pathology and fibrosis of the lung, inhibiting the positive feedback loop of MIF/NF-*κ*B, and reducing lymphocyte homing to bronchial mucosa. This model revealed the immune mechanism of UC-related lung injury and the intervention mechanism of the Chinese medicine, which provided the rationale for treating ulcerative colitis clinically, so as to demonstrate the theory of “the lung and the large intestine being interior-exteriorly related” and “treating the same disease with different approaches.”

## 1. Introduction

Traditional Chinese medicine (TCM) has a long history for thousands of years. Its origin can be traced back to remote antiquity. In a long course of struggling against diseases, TCM evolved into a unique and integrated theoretical system of TCM. The theoretical system takes the physiology and pathology of zang-fu organs and meridians as its basis and treatment based on syndrome differentiation (TDS) as its diagnostic and therapeutic features. As for the relationship between “disease” and “treatment,” TCM takes two different clinical ways on the basis of TDS. One is “treating the same disease with different therapies,” which means that the same disease may manifest itself in different syndromes at different stages or under different conditions. Therefore, the therapies for the same disease should be adopted towards different therapies according to the patient's constitution, the geographical environment, and the climatic and seasonal changes. The principle of “treating the same disease with different approaches” has a long history. It was first seen in *Huangdi Neijing*. However, for the same disease, its pathogenesis and treatment are different, which also belongs to the principle of “treating the same disease with different approaches.” “The lung and the large intestine being interior-exteriorly related” is one of the most representative theories in traditional medicine, which embodies the systematic and holistic view of disease cognition in traditional Chinese medicine. In clinical practice, the theory of “the lung and the large intestine being interior-exteriorly related” reflects the intestinal origin theory of lung disease, and it is also the theoretical basis for the intestinal treatment of lung disease. In traditional Chinese medicine, “the lung and the large intestine being interior-exteriorly related” participates in human life activities through the interaction of collaterals, Qi mechanism, water, fluid metabolism, and so on. *Lingshu meridians* show that “Taiyin-lung channels start from the middle Jiao, the lower collateral large intestine. The upper diaphragm belongs to the lung,” “Yangming-large intestine channels start from the end of the big finger... The collateral lung and the lower diaphragm belongs to the large intestine.” It shows that the lung and large intestine are connected with each other through meridians. The pathological changes in the lung can be treated by both lung meridian drugs and intestinal meridian drugs, which fully reflects the traditional theory of “treating the same disease with different approaches” and further verifies the theoretical basis of “the lung and the large intestine being interior-exteriorly related”.

The incidence of ulcerative colitis (UC) which is a chronic, relapsing, and unknown etiology inflammatory bowel disease is on the increase worldwide. Typical symptoms of UC include acute pain, diarrhea with or without mucus and blood, and extraintestinal manifestations [1]. It is classified as a refractory disease by the World Health Organization (WHO). The extraintestinal manifestations of UC involve the lung, mouth, skin, and other organs, and they develop one or more symptoms expressed as a chief complaint. A significant fraction of the patients with frequent extraintestinal manifestations present with symptoms of pulmonary dysfunction and lung injury. At present, a large number of studies have been carried out that lung and bronchus injuries are as important extraintestinal manifestations with an incidence rate of up to 50% in China and abroad. In the 1970s, Kraft et al. [2]were the first to report that inflammatory bowel disease could involve the lung. In the following 40 years, there were many reports about lung injury or inflammatory bowel disease. In modern medicine, much research on a close correlation between the lung and bowel elaborated from embryonic development [3], mucosal biofilms [4], and mucosal immune [5]. From the perspective of the mucosal immune system: both gastrointestinal and respiratory mucosa is part of the public mucosal immune system. When one mucosal lesion occurs, it can affect the other through the mucosal immune pathway. The hypothesis from Aydin Yilmaz [6] supported the relationship between respiratory damage of IBD and pathophysiological mechanism. Both colonic and respiratory epithelial cells contain goblet cells and submucous glands; moreover, the common submucosal lymphoid tissues of the lung and gastrointestinal tract play an important role in the host's mucosal defense system. The high similarity of the mucosal immune system is the cause of pathological similarity. In the clinical practice of TCM, UC-related lung diseases are treated both from the lung and the large intestine, which reflects the TCM thought of “the lung and the large intestine being interior-exteriorly related” and “treating the same disease with different approaches.”

Chinese traditional medicine has a long history of thousands of years. It inherits the valuable experience and theoretical knowledge of the ancient people in fighting against various diseases. Modern medical research elaborates the mechanism of TCM in treating various diseases in detail. It has been reported that the extract of methanol leaf of orchid can have significant neuropharmacological and antidiabetes properties [7]. Enodin has a wide range of pharmacological activities, especially in neuroprotection [8]. Narirutin, a component in citrus fruits, has several pharmacological properties such as anticancer activity, neuroprotection, stress relief, liver protection, antiallergic activity, antidiabetes activity, antilipogenic activity, antiobesity effect, and immune regulation [9]. There are also reports showing that Citrus limon extracts have neuropharmacological properties [10]. Cruciferous vegetables and their important bioactive metabolites can significantly prevent and treat colorectal cancer [11]. In addition, there are many plants or herbs with a certain ability to prevent or treat diseases, such as Andrographis paniculata [12], Lepidagathis hyalina [13], Ophiorrhizarugosa leaves [14], coumarin [15, 16], and curcumin [17]. In this study, we chose Huangqi Jiegeng decoction which was attributed to the lung channel and Huangqi Huanglian decoction which was attributed to the intestine channel separately for treating UC-related lung injury and found that both large intestine and pulmonary drugs could effectively treat lung injury caused by ulcerative colitis, which further verified the basic theory of “the lung and the large intestine being interior-exteriorly related” and the therapeutic theory of “treating the same disease with different approaches.” It contributes to realize the importance of the prevention and early intervention of UC-related lung damage and opens up a new way to solve the problem of refractory UC fundamentally.

## 2. Materials and Methods

### 2.1. The Information on Traditional Chinese Medicine

To mimic the traditional route of administration, the traditional Chinese Medicine was suspended in distilled water and given to the animals intragastrically using a feeding tube. Huangqi Jiegeng decoction (Table 1) and Huangqi Huanglian decoction (Table 2) consist of 13 Chinese herbal medicines, respectively. These two compounds' decoction-free granules were all purchased in Dongzhimen Hospital (Beijing), dissolved in water at 70°C for 30 mins, and stored at −20°C. Western medicine control (Sulfasalazine, lot number is H31020450) was produced by Shanghai Sanwei Pharmaceutical Co., Ltd., stored at −20°C after water dissolution.

### 2.2. Animals

Male Wistar rats weighing 200 ± 10 g were purchased from the Academy of Military Medical Laboratory Animal Centre (Beijing, China). Ten male New Zealand rabbits weighing about 3 kg were purchased from Haidian Thriving Animal Farm (Beijing, China). All animals were housed at SPF Animal Laboratory of Dongzhimen Hospital (Beijing, China) with free access to food and water and kept in a regulated environment (23 ± 2°C) under a 12-hour light/dark cycle (with light turning on at 8: 00 am). All animal procedures were performed strictly within national regulations and guidelines of the National Institutes of Health (NIH) and approved by the Animal Experimentation Committee at the Beijing University of Chinese Medicine.

### 2.3. Induction of Ulcerative Colitis and the Chinese Medicine

Antigen preparation: ten rabbits were killed by CO_2_ suffocation, and then the colon was removed immediately and rinsed with sterile saline, and scraped the mucosa. The mucosa was mixed with equal saline and homogenized 30 times with a tight Dounce homogenizer (Sigma, USA). Samples were further disrupted by intermittent sonication (six 30 s pulse with a 1 min cooling period in between) and then centrifuged at 3,000 rpm (Eppendorf, Germany) for 30 mins at 4°C. The supernatant was then aliquoted and stored at −20°C. The protein concentration was measured by a bicine cholinic acid (BCA) assay (CoWin Bioscience, China).

Antigen preimmunization and TNBS enema: rabbit intestinal mucosal antigen solution was mixed with an equal volume of Freud's complete adjuvant, which was preparing for the antigen emulsion. Wistar rats were immunized with the antigen emulsion in the paws and groin alternately on day 1, day 15, and day 22. Each immune volume contained 8 mg of antigen protein per rat. On day 29, a medical-grade polyurethane cannula for enteroclysm (external diameter 2 mm) was inserted into the anus, and the tip was advanced to 8 cm proximal to the anal verge. TNBS (Sigma, USA) dissolved in 50% ethanol was instilled into the colon rapidly with TNBS 100 mg/kg (0.5–0.7 ml per rat). Then the rats were maintained in a head-down position for one minute to prevent leakage of the intraintestinal instillation. The rats alive were randomly divided into seven groups after TNBS-alcohol enema, and the rats with ulcerative colitis received an intragastric administration with Traditional Chinese Medicine. All the experimental rats were killed by CO_2_ asphyxiation within 1 week and 5 weeks respectively.

### 2.4. The Histopathological of Lung, Bowel, Liver, and Kidney, and the Fibrotic Changes of Lung and Bowel Were Observed

The lung, bowel, liver, and kidney of the rats were taken and soaked in a 4% paraformaldehyde solution. The 4% paraformaldehyde solution was changed every day. One week later, the fixed specimens were routinely dehydrated with alcohol gradient, transparent xylene, embedded with paraffin, and sectioned. HE staining and Masson staining were performed, and photos were taken under the light microscope.

### 2.5. Radioimmunoassay Analysis and ELISA

Blood was drawn from the abdominal aorta, the blood serum was deep frozen in liquid nitrogen, and all rats were killed by CO_2_ suffocation. The lung tissue was also taken off, washed with normal saline, absorbed the water with filter paper, and deep frozen in liquid nitrogen. When used, add 5 times of water into the lung, disrupt the lung tissue with ultrasonic disintegrator by intermittent sonication (six 30 s pulse with a 1 min cooling period in between), and then centrifuge the sample at 3,000 rpm for 20 mins at 4°C. The supernatant was collected, and TNF-a and IL-8 in lung tissue of rats in each group were detected with a radioimmunity kit (Beijing Kangyua Ruide Biotechnology Co. Ltd.), and the MadCAM-1 in the serum was detected with ELISA kit (Beijing Kangyua Ruide Biotechnology Co. Ltd.).

### 2.6. Real-Time PCR Analysis

The total RNA was extracted using the TRZol reagent extraction kit (Invitrogen Life Technologies, Inc). The mRNA expressions of TLR4, NF-*κ*B, MIF, MadCAM-1, and GAPDH in each group were detected by real-time PCR. The sequences of the PCR primers are shown in Table 3. Ct of every sample was analyzed by MxPro-Mx3000p software. The relative amount of each gene was calculated by utilizing the expression of GAPDH as an internal control by using equation 2△△Ct where ΔCt = (Ct gene-Ct GAPDH). △△Ct ＝ △Ct － average (△Ct normal), cDNA ＝ 2△△Ct. All real-time PCR experiments were performed with Power SYBR Green PCR Master Mix (Applied Biosystems company, USA).

### 2.7. Immunohistochemistry Analysis

To demonstrate the expression and localization of IL-8 and TNF-*α*, we used immunohistochemistry to detect. The tissue sections of rats in each group were incubated with IL-8 (antirabbit, 0.1 mg/ml, Abcam) or TNF-*α* (antirabbit, Abcam) and detected, respectively, with the secondary antibodies (CoWin Bioscience, China).

### 2.8. Western Blot Analysis

The tissue was then lysed with 200 *μ*l RIPA lysis buffer. Protein contents were quantitated using a BCA protein reagent assay kit (CoWin Bioscience, China) and analyzed by 10–12% of SDS-PAGE, followed by immunoblotting using enhanced chemiluminescence substrate (Merck Millipore) according to the manufacturer's instructions. The protein expressions of IL-10 in the lung were detected by Western Blotting. Bands were visualized using a chemiluminescent detection system (ProteinSimple, San Jose, CA, USA).

### 2.9. Statistical Analysis

Quantitative data were expressed as means ± standard deviation (s.d.). The significant difference between groups was assessed using Student's *t*-test and one-way ANOVA. Post hoc comparisons were made using the nonparametric Dunn multiple comparison test. In all tests, the criterion for statistical significance was *P* < 0.05. Statistical analysis was performed with SPSS Software 13.0.

## 3. Results

### 3.1. The Protective Effect of Traditional Chinese Medicine on Viscera

After 4 weeks of administration, the colon tissue structure of the normal group was intact, the intestinal mucosa was normal, and there was no inflammatory cell infiltration. In the model group, there were extensive lymphocytic inflammatory infiltration, necrosis of the colon wall, and a large number of ulcers (Figure 1(a)). The structure of the lung tissue, alveolar, and bronchioles was normal and clear with no inflammatory cell infiltration or fibrosis hyperplasia in the normal group. In the model group, there were extensive lymphocytic infiltration and narrow alveoli. Each treatment group improved with differing degrees of pathological changes and fibrosis. However, there was still a lot of inflammatory infiltration with lymphocytes in the SASP group and HQHLD group (Figure 1(b)). Masson's staining visualized substantial collagen tissue existed on the intestinal mucosal ulcer surface and intestinal mucosal basement in the model group, even replacing normal mucosa and glands (Figure 1(c)). There was a dense hyperproliferation of collagen tissues around the bronchial tissues of the model group, more than that in the normal group. The collagen tissue hyperproliferation in each treatment group was more than in the normal group, but lighter than in the model group significantly (Figure 1(d)).

### 3.2. Traditional Chinese Medicine Groups Downregulated the Expression of TLR4, NF-Κb, and MIF

After 4 weeks of administration, the model group had a higher level of TLR4 mRNA expression than the normal group (*P* < 0.01). The expression of TLR4 mRNA in the SASP group and HQHLD group was obviously increased compared with the normal group (*P* < 0.01; *P* < 0.05), and all Chinese Medicine treatment groups were lower than the model control group (*P* < 0.05) (Figure 2(a)). The levels of NF-*κ*B mRNA expression were increased in the model group compared with the normal group, and this difference was shown to be significant (*P* < 0.05). The expression of NF-*κ*B mRNA in all treatment groups was obviously decreased compared with the model group (*P* < 0.01, *P* < 0.05) (Figure 2(b)). The model group had a significantly higher level of MIF mRNA expression than the normal group (*P* < 0.001); the expression of MIF mRNA in all treatment groups was obviously decreased compared with the model group (*P* < 0.01). MIF mRNA expression in the SASP group was obviously lower than that in the normal group (*P* < 0.05) (Figure 2(c)). These results suggested that the increase of TLR4 gene transcription activation and NF-*κ*B expression may have been the cause of lung injury in 4 weeks chronic inflammatory phase of this UC model. Each treatment group could reduce lung injury by decreasing the transcription activation of the TLR4 gene and the expression of NF-*κ*B. Compared with the model group, the expression of MIF mRNA in all treatment groups was significantly decreased, which indicated that as in the SASP group, all Chinese medicine groups could alleviate pulmonary inflammation by decreasing macrophage infiltration into lung tissues.

### 3.3. Traditional Chinese Medicine Groups Decreased the Expression of TNF-A and IL-8

After 4 weeks of administration, radioimmunoassay showed the model group had a higher level of IL-8 expression than the normal group (*PP* < 0.05), and the expression of IL-8 in all treatment groups was obviously decreased compared with the model group (*P* < 0.01); however, no significant difference was found comparing with the normal group (Figure 3(a)). The model group had a significantly higher level of TNF-*α* (Figure 3(c)) and IL-6 (Figure 3(e)) expression than the normal group (*P* < 0.001), and the expression level of TNF-*α* and IL-6 in lung tissue of HQJGD group and HQHLD group was significantly lower than that of the model group (*P* < 0.05). Immunohistochemistry also showed that IL-8 (Figure 3(b)), TNF-*α* (Figure 3(d)), and IL-6 (Figure 3(f)) were decreased in each treatment group. The results showed that the chemotaxis and activation of neutrophils were enhanced in the model group, and the lung injury caused by neutrophils in each treatment group had a certain therapeutic effect. The above results showed that the HQJGD group and HQHLD group could reduce the expression of TNF-*α* and IL-6, and each treatment group had a certain therapeutic effect on lung injury caused by IL-8.

### 3.4. Traditional Chinese Medicine Groups Decreased the Expression of MAdCAM-1 mRNA

After 4 weeks of administration, the model group had a significantly higher level of MAdCAM-1 mRNA expression than the normal group (*P* < 0.001), the expression level of MAdCAM-1 mRNA in lung tissue of all Chinese Medicine treatment groups was significantly lower than that of the model group (*P* < 0.01), and no significant difference was found comparing with the normal group (*P* > 0.05). The expression level of MAdCAM-1 mRNA in the SASP group was significantly higher than that in the normal group (*P* < 0.01) and lower than that in the model group (*P* < 0.01) (Figure 4). The above results showed that after 4 weeks of administration, all Chinese medicine groups could decrease the expression of MAdCAM-1 mRNA in the lung compared with the model group, which indicated that as in the SASP group, all Chinese medicine groups could alleviate pulmonary inflammation by reducing lymphocyte homing to bronchial mucosa.

### 3.5. Perfect Specificity in UC-Related Lung Injury

The weight of the model group rats decreased significantly compared to that of the normal group rats after 4 weeks of drug administration (*P* < 0.01) (Figure 5(a)). The results showed that the weight of rats decreased after modeling and increased after administration. There was no significant difference in serum ALT and AST (*P* > 0.05) (Figure 5(b)). Within 4 weeks of administration, the serum BUN of the SASP group was significantly lower than that of the model group (*P* < 0.01), and there was no significant difference in other groups (*P* > 0.05). There was no significant difference in serum creatinine (CR) between each group (*P* > 0.05) (Figure 5(b)). After 4 weeks of administration, the pathological morphology of the liver in each group was basically normal, the structure of the hepatic cord was clear, the hepatocytes were arranged radially with the central vein as the center, and there was no fat vacuole in the liver tissue. The structure of the liver lobule was intact, the arrangement of liver cells was normal, a few Oliver cells appeared apoptosis and fatty degeneration, the fibrous tissue did not hyperproliferate obviously, and the necrosis of liver cells in the SASP group was slightly more than that in other groups (Figure 5(c)). Basically, there is normal pathological morphology of renal tissue in each group. Hyperplasia or necrosis in glomerular cells and mesangial matrix has not been seen yet, and no lesions were revealed in tubuloinsterstitial and renal vessels (Figure 5(d)). The results above showed that lung injury induced by UC had perfect specificity. “The lung and the large intestine being interior-exteriorly related” theory was further verified.

## 4. Discussion

Based on our previous research, an immune-TNBS-ethanol rat model was established. The pathological changes in the lung, intestine, liver, and kidney were observed; cytokines, chemokines, and adhesion molecules in lung tissue were detected in order to explore the immunological mechanism of lung injury in UC rats, and the results showed that intestinal lesions can cause lung damage specifically. We found that except for the Chinese medicine Huangqi Jiegeng Decoction which was attributed to lung meridian, HQHLD attributed to intestinal meridian could also improve the UC-related lung injury, which indicates the internal relationship between the lung and the large intestine, so as to laterally verify the theory of viscera related to “the lung and the large intestine being interior-exteriorly related” and “treating the same disease with different therapies”; it will lay a solid theoretical foundation for the clinical treatment of lung and intestinal diseases in the future. In addition, the treatment of traditional Chinese medicine did not cause any damage to the liver and kidneys.

Toll-like receptors (TLRs) are the pattern recognition receptors of IECs intestinal innate immune system for the recognition of pathogen-associated molecular patterns (PAMPs) [18] in the intestinal lumen. It is mainly responsible for monitoring the microecological balance in the enteric cavity and transmitting that information to the lamina propria cells of the mucous membrane [19]. Under normal circumstances, the expression of TLR4 is extremely sparse. However, TLR4 is abundantly expressed in epithelial cells and lamina propria cells of colon mucosa in UC patients [20]. When TLR4 ligand such as LPS binds to TLR4 of abnormal expression, NF-*κ*B was activated through MyD88, the primary immune response protein of bone marrow differentiation [21, 22]. Activation of NF-*κ*B can regulate the expression of many inflammatory molecules related to IBD, including TNF-*α*, IL-6, IL-8, ICAM1, and other activating factors and adhesion molecules [23, 24]. The increased inflammatory factors can directly injure the intestinal mucosa or induce TLR4-positive macrophages recruitment to the inflammatory mucosa. At the same time, the antigenic material in the intestinal lumen directly into the epithelial cells passes through the damaged mucosal barrier, further exacerbating the inflammatory response [25].

Macrophage migration inhibitory factor (MIF) is the first cytokine with multiple effects on inflammatory mediators function. MIF is involved in multiple pathophysiological processes such as inhibiting the migration of activated macrophages, activating lymphocytes, killing tumor cells, inducing macrophages to secrete a variety of proinflammatory factors, and inhibiting the anti-inflammatory effect of glucocorticoids [26]. It is an important regulator of innate immunity and acquired immunity. The production and release of MIF are regulated by multiple factors. Cytokine TNF-*α* can stimulate monocyte/macrophage to release MIF. MIF plays an important role in the occurrence and development of inflammatory diseases such as sepsis and acute respiratory distress syndrome [27, 28]. In patients with ulcerative colitis, MIF may induce mucosal damage by promoting macrophage infiltration in local intestinal mucosa and inducing macrophage to produce IL-8. In addition. MIF can upregulate the expression of TLR4. MIF can activate the TLR4 gene by the ETS family member PU.1, which encodes receptor complex binding to LPS. TLR4 activates NF-*κ*B, causes macrophages to activate, proliferates, and releases inflammatory factors. TLR4 plays an important role in innate immunity. MIF and NF-*κ*B can form a positive feedback loop. Many inflammatory factors, such as TNF-*α*, IL-1*β* [29], and ox LDL [30], can promote the release of MIF through this pathway. As shown in the above study, the relationship between MIF and each pathway is not isolated but exists in the form of the regulatory network.

Our study showed that the TLR4 receptor and its mediated NF-*κ*B signaling in lung tissue of the model group may be an important link in the pathogenesis of lung injury caused by UC. The partial elucidation of the TLR4/NF-*κ*B pathway provides a new opportunity for the treatment of UC-related lung injury. Each treatment group can reduce lung injury by downregulating the expression of the TLR4 gene and NF-*κ*B in lung tissue. In addition, in the positive feedback loop formed by MIF and NF-*κ*B, the expression of MIF was significantly reduced in each treatment group. The expression of TNF-*α*, IL-8, and IL-6 was increased in the lung of the model group, and the expression of TNF-*α* was decreased to a certain extent by HQJGD and HQHLD. All the treatment groups were able to significantly reduce the expression of IL-8, suggesting that each treatment group had a certain therapeutic effect on the lung injury caused by the positive feedback pathway of MIF and TLR4/NF-*κ*B. Among them, HQHLD which was attributed to the intestine meridian could significantly reduce the expression of MIF and TLR4/NF-*κ*B positive feedback pathway in pulmonary inflammation, which embodies the “Treatment of lung disease from intestines” and “Treating the same disease with different therapies,” and further clarifies the material basis of TCM theory of “the lung and the large intestine being interior-exteriorly related.”

Mucosal addressin cell adhesion molecule-1 (MAdCAM-1) belongs to the member of the immunoglobulin superfamily. It is an adhesion molecule selectively expressed on the surface of vascular endothelial cells of the intestinal mucosa and related lymphoid tissues, which mediates primarily the selective homing of lymphocytes to normal mucosa [31]. The adhesion mechanism of MAdCAM-1 plays an important role in the gut mucosal-associated lymphoimmune system. Clinical and animal experimental studies have confirmed that UC is associated with the abnormal expression of MAdCAM-1, and the expression of MAdCAM-1 in vascular endothelial cells of the inflamed colon in UC patients is upregulated. IL-1 and TNF-*α* can induce the expression of MAdCAM-1 in mouse epithelial cells [32]. Kato et al. [33] found the expression of MAdCAM-1 significantly increased with a prolonged time in DSS-induced colitis in mice, and there were a large number of integrin and lymphocyte gathering into the colitis site, suggesting that MAdCAM-1 was the main inducible factor which mediates lymphocyte migration to the inflammatory colonic mucosa. MAdCAM-1 is an important molecule involved in the local homing of lymphocytes. Under normal conditions, MAdCAM-1 is barely expressed in the human lung but appears in our UC model, which clarifies the specific correlation between the lung and large intestine. Each treatment group alleviated the lymphocyte homing into the pulmonary and bronchial mucosa, and the interventions of HQJGD were the most significant. Meanwhile, HQHLD attributed to intestine meridian effectively inhibited lymphocyte homing into pulmonary, improved the UC-related lung inflammation, and further provided the basis for the TCM theory of “the lung and the large intestine being interior-exteriorly related” and “treating the same disease with different therapies.”

## 5. Conclusions

In conclusion, although the pathogenesis of UC-related lung injury has not been fully elucidated, immune factors are of great significance. In this article, we have made a start on the TCM theory of “the lung and the large intestine being interior-exteriorly related,” attempted to establish the animal experimental model based on “Lung injury induced by enteropathy,” and treated UC-related lung injury with the theory of “treating the same disease with different therapies,” so as to simulate the relationship between lung and intestine of the human body. Through animal models, we found that the Chinese medicine Huangqi Jiegeng Decoction attributed to lung meridian and the Chinese medicine Huangqi Huanglian Decoction attributed to intestine meridian could alleviate pulmonary inflammation in UC-related lung injury by obviously improving the pathology and fibrosis of the lung, inhibiting the positive feedback loop of MIF/NF-Κb and reducing lymphocyte homing to bronchial mucosa, so as to elaborate the theory of “the lung and the large intestine being interior-exteriorly related” (Figure 6). Although these animal models in this study could produce symptoms and intestinal pathological changes close to UC clinically, and lesions could have a long maintenance time and good reproducibility, there were also a long-time modeling with the tedious operation and a certain mortality rate. Thus, the method of modeling needs to be further improved in the next study.

## Figures and Tables

**Figure 1:** Pathological and fibrosis changes of lung and bowel tissues in rats with ulcerative colitis. UC models were established with the mucous membrane of colon allergize combined with TNBS-alcohol enteroclysis. (a) Bowel tissues with HE staining. (b) Lung tissues with HE staining. (c) Bowel tissues with Ma Song dyeing. (d) Lung tissues with Ma Song dyeing. 1 (4w normal), 2 (4w model), 3 (SASP group), 4 (HQJGD group), and 5(HQHLD group).

**Figure 2:** The expression of TLR4 mRNA, NF-*κ*B mRNA, and MIF mRNA in the UC-related lung injury tissues. UC models were established with the mucous membrane of colon allergize combined with TNBS-alcohol enteroclysis. (a) TLR4 mRNA. (b) NF-*κ*B mRNA. (c) MIF mRNA. Compared with the normal group,  ^*∗*^*P* < 0.05;  ^*∗*^ ^*∗*^*P* < 0.01;  ^*∗*^ ^*∗*^ ^*∗*^*P* < 0.001. Compared with the model group, #*P* < 0.05, ##*P* < 0.01.

**Figure 3:** The expression of TNF-*α* and IL-8 in the UC-related lung injury tissues. UC models were established with the mucous membrane of colon allergize combined with TNBS-alcohol enteroclysis. (a) The expression of IL-8 (radioimmunoassay). (b) The expression of IL-8 (Immunohistochemistry). (c) The expression of TNF-*α* (Radioimmunoassay). (d) The expression of TNF-*α* (Immunohistochemistry). (e) The expression of IL-6 (RT-PCR). (f) The expression of IL-6 (immunohistochemistry). 1 (4w normal), 2 (4w model), 3 (SASP group), 4 (HQJGD group), and 5 (HQHLD group). Compared with the normal group,  ^*∗*^*P* < 0.05;  ^*∗*^ ^*∗*^*P* < 0.01;  ^*∗*^ ^*∗*^ ^*∗*^*P* < 0.001. Compared with the model group, #*P* < 0.05, ##*P* < 0.01.

**Figure 4:** The expression of MAdCAM-1 mRNA in the UC-related lung injury tissues. UC models were established with the mucous membrane of colon allergize combined with TNBS-alcohol enteroclysis. MAdcam-1 mRNA expression in the lung (RT-PCR). Compared with the normal group,  ^*∗*^*P* < 0.05;  ^*∗*^ ^*∗*^*P* < 0.01;  ^*∗*^ ^*∗*^ ^*∗*^*P* < 0.001. Compared with the model group, #*P* < 0.05, ##*P* < 0.01.

**Figure 5:** Perfect specificity in UC-related lung injury. Ulcerative colitis models were established with mucous membranes of colons sensitized with TNBS-alcohol enteroclysis. (a) Body weight changes. (b) Hepatorenal function changes. ALT, AST, BUN, and Cr were evaluated. HE staining of the liver (c) and kidney (d). 1 (4w normal), 2 (4w model), 3 (SASP group), 4 (HQJGD group), and 5 (HQHLD group). Compared with the normal group,  ^*∗*^*P* < 0.05;  ^*∗*^ ^*∗*^*P* < 0.01;  ^*∗*^ ^*∗*^ ^*∗*^*P* < 0.001. Compared with the model group, #*P* < 0.05; ##*P* < 0.01.

**Figure 6:** Huangqi Jiegeng decoction attributed to lung meridian and Huangqi Huanglian decoction attributed to intestine meridian could effectively improve the lung injury induced by UC by inhibiting the positive feedback loop of MIF/NF-*κ*B, so as to elaborate the theory of “the lung and the large intestine being interior-exteriorly related.”

**Table 1:** Composition of Huangqi Jiegeng decoction.

Chinese medicinal plant	Latin name	Batch number	Weight (g)
*Astragalus membranaceus (Fisch.)*	*Astragalus membranaceus (Fisch.) Bunge*	19071411	30
*Platycodi Radix*	*Platycodon grandiflorum (Jacq.) A.DC.*	19091931	6
*P. veitchii Lynch*	*Paeonia veitchii Lynch*	19040411	10
*Paeonia Lactiflora Pall*	*Paeonia lactiflora Pall.*	19070321	10
*Aurantii fructus*	*Citrus aurantium L.*	19111971	10
*Galla chinensis*	*Rhus chinensis Mill.*	19020211	6
*Licorice*	*Glycyrrhiza glabra L.*	19102121	10
*Pericarpium Citri Reticulatae*	*Citrus reticulata Blanco*	20010881	10
*Saposhnikovia divaricata*	*Saposhnikovia divaricata (Turcz.) Schischk.*	20010341	10
*Forsythia suspensa*	*Forsythia suspensa (Thunb.) Vahl*	18121591	12
*Coix seeds*	*Coix lacryma-jobi L. var. Mayuen (Roman.) Stapf*	19090431	30
*Bletilla striata*	*Bletilla striata (Thunb.) rchb. f.*	18121031	10
*Scutellaria Baicalensis*	*Scutellaria baicalensis Georgi*	19061431	10

**Table 2:** Composition of Huangqi Huanglian decoction.

Chinese medicinal plant	Latin name	Batch number	Weight (g)
*Astragalus membranaceus*	*Astragalus membranaceus (Fisch.) Bunge*	19071411	30
*Coptis chinensis*	*Coptis chinensis Franch.*	19080711	10
*P. veitchii Lynch*	*Paeonia veitchii Lynch*	19040411	15
*Paeonia lactiflora Pall*	*Paeonia lactiflora Pall.*	19070321	15
*Aucklandia lappa Decne*	*Aucklandia lappa Decne.*	19093041	6
*Galla chinensis*	*Rhus chinensis Mill.*	19020211	6
*Licorice*	*Glycyrrhiza glabra L.*	19102121	6
*Panax notoginseng*	*Panax notoginseng (Burk.) F. H. Chen*	19021161	3
*Atractylodes macrocephala*	*Atractylodes macrocephala Koidz.*	19082551	10
*Areca nut*	*Areca catechu L.*	19061031	10
*Sanguisorba officinalis L*	*Sanguisorba officinalis L.*	19051651	15
*Dandelion*	*Taraxacum borealisinense Kitam.*	19081521	20
*Coix seeds*	*Coix lacryma-jobi L. var. Mayuen (Roman.) Stapf*	19090431	20

**Table 3:** PCR primer(s)

Gene	Sequence of primers (5′-3′)	Product size	Cycling parameters
TLR4	F: CTT TCA GGG AAT TAG GCT CC R: CCA AGA TCA ACC GAT GGA C	116 bp	10 min at 95°C, 30sec at 95°C, 30sec at 55°C, 20 sec at 72°C, for 40 cycles
NF-*κ*b	F: ATC TGT TTC CCC TCA TCT T R: GTG CGT CTT AGT GGT ATC TG	167 bp	10 min at 95°C, 30sec at 95°C, 30sec at 55°C, 20 sec at 72°C, for 40 cycles
MIF	F: TCT CCG CCA CCA TGC CTA TG R: GGG TCG CTC GTG CCA CTA AA	178 bp	10 min at 95°C, 30sec at 95°C, 30sec at 60°C, 20 sec at 72°C, for 40 cycles
MAdCAM-1	F: CCG AAA TCC ACC AGA ACC R: TCC AAT GCA CCG TCA CTC	81 bp	10 min at 95°C, 30sec at 95°C, 30sec at 54°C, 20 sec at 72°C, for 40 cycles
GAPDH	F: CCA TGG AGA AGG CTG GG R: CAA AGT TGT CAT GGA TGA CC	195 bp	10 min at 95°C, 30sec at 95°C, 30sec at 54°C, 20 sec at 72°C, for 40 cycles

## Data Availability

The data and materials in this study are available from the corresponding author upon reasonable request.

## Abbreviations

UC: Ulcerative colitis
IBD: Inflammatory bowel disease
TNBS: 2,4,6-Trinitrobenzenesulfonic acid
ALT: Alanine aminotransferase
AST: Aspartate aminotransferase
BUN: Blood urea nitrogen
Cr: Serum creatinine
SASP: Sulphasalazine
HQJGD: Huangqi Jiegeng decoction
HQHLD: Huangqi Huanglian decoction
TLR4: Toll-like receptor 4
NF-*κ*B: Nuclear factor kappa-B
MIF: Macrophage migration inhibitory factor
TNF-*α*: Tumor necrosis factor-*α*
IL-6: Interleukin-6
IL-8: Interleukin-8
MAdCAM-1: Mucosal addressin cell adhesion molecule-1
TCM: Traditional Chinese medicine.
